# Isoflurane Preconditioning Confers Cardioprotection by Activation of ALDH2

**DOI:** 10.1371/journal.pone.0052469

**Published:** 2013-02-28

**Authors:** Xiao-E Lang, Xiong Wang, Ke-Rang Zhang, Ji-Yuan Lv, Jian-Hua Jin, Qing-Shan Li

**Affiliations:** 1 Department of Cardiology, The First Clinical Medical College of Shanxi Medical University, Taiyuan, Shanxi, China; 2 Department of Psychiatry, The First Clinical Medical College of Shanxi Medical University, Taiyuan, Shanxi, China; 3 Department of Nuclear Medicine, The First Clinical Medical College of Shanxi Medical University, Taiyuan, Shanxi, China; 4 School of Pharmaceutical Science, Shanxi Medical University, Taiyuan, China; National Cancer Institute, United States of America

## Abstract

The volatile anesthetic, isoflurane, protects the heart from ischemia/reperfusion (I/R) injury. Aldehyde dehydrogenase 2 (ALDH2) is thought to be an endogenous mechanism against ischemia-reperfusion injury possibly through detoxification of toxic aldehydes. We investigated whether cardioprotection by isoflurane depends on activation of ALDH2.Anesthetized rats underwent 40 min of coronary artery occlusion followed by 120 min of reperfusion and were randomly assigned to the following groups: untreated controls, isoflurane preconditioning with and without an ALDH2 inhibitor, the direct activator of ALDH2 or a protein kinase C (PKCε) inhibitor. Pretreatment with isoflurane prior to ischemia reduced LDH and CK-MB levels and infarct size, while it increased phosphorylation of ALDH2, which could be blocked by the ALDH2 inhibitor, cyanamide. Isolated neonatal cardiomyocytes were treated with hypoxia followed by reoxygenation. Hypoxia/reoxygenation (H/R) increased cardiomyocyte apoptosis and injury which were attenuated by isoflurane and forced the activation of ALDH2. In contrast, the effect of isoflurane-induced protection was almost abolished by knockdown of ALDH2. Activation of ALDH2 and cardioprotection by isoflurane were substantially blocked by the PKCε inhibitor. Activation of ALDH2 by mitochondrial PKCε plays an important role in the cardioprotection of isoflurane in myocardium I/R injury.

## Introduction

Acute myocardial infarction (AMI) is responsible for the death of millions of persons worldwide each year [1]. Murry et al. demonstrated that a succession of short periods of myocardial ischemia and reperfusion prior to the continuous maintenance of coronary reperfusion protects the myocardium against subsequent prolonged ischemic insults, which has been termed ‘ischemic preconditioning’ (IPC) [2]. This phenomenon is achieved by several pharmacological agents, including volatile anesthetics. Volatile anesthetics such as isoflurane have cardioprotective effects when administered before a period of myocardial ischemia and reperfusion, and this phenomenon is referred to as anesthetic preconditioning (APC) [3], [4]. APC is a cardioprotective strategy that increases resistance to ischemia and reperfusion (I/R) by eliciting innate protective mechanisms, and was described in various animal models [3]–[6], as well as in humans [7], [8]. APC has been shown to reduce infarct size, and attenuate contractile dysfunction and serum CK-MB concentration caused by myocardial ischemia. Cellular signaling during APC is complex, and in many aspects, comparable to that of IPC. The intracellular mechanisms involved in APC have not been completely identified. It has become clear that multiple cellular pathways participate in the establishment of a cellular phenotype that makes the heart more resistant to ischemic damage. Mechanisms reported to date involve inhibition of mitochondrial permeability transition pore (mPTP) opening [9], the activation of kinases such as protein kinase C (PKC) [10], [11], the generation of reactive oxygen species (ROS) [12], [13], and opening of adenosine triphosphate-sensitive potassium channels (K_ATP_) [3], [14], [15] ^.^

Translocation of PKC isoforms from the cytosol to the membranes is known to be a key mediator in IPC. PKC epsilon (PKCε) activation is required and is sufficient to protect the heart from ischemia and reperfusion (I/R) injury [16], [17]. Recent evidence suggests that PKCε is targeted to the mitochondria and interacts with many mitochondrial proteins, including mitochondrial aldehyde dehydrogenase 2 (ALDH2) [18]. The mitochondrial isoform of ALDH2 plays a key role in the metabolism of acetaldehyde and other toxic aldehydes, whose phosphorylation and activation by PKCε is required to confer cardioprotection [19], [20]. Overexpression of the ALDH2 transgene alleviates I/R injury, post-I/R and ischemic ventricular dysfunction [21], [22]. Consistent with this, ALDH2 knockout exacerbated I/R injury [23]. These data support the essential role of ALDH2 against I/R injury in the heart. Nonetheless, the mechanism(s) behind ALDH2-induced protection against I/R injury may be diverse, involving bioactivation of nitroglycerin, and reducing the production of free radicals [24], and ultimately mitochondrial dysfunction [23], all hallmarks of I/R injury. As anesthetic-induced preconditioning can also be demonstrated in humans, a thorough understanding of the signal transduction involved might have an impact on the clinical applicability of cardioprotection by APC. However, the role of ALDH2 in isoflurane-induced APC has not been investigated. Thus, the current study tested the hypothesis that PKCε-mediated activation of mitochondrial ALDH2 plays a critical role in isoflurane preconditioning.

## Materials and Methods

### Animals

Male Sprague-Dawley (SD) rats, weighing 200–220 g, were used in this study. The animals were provided by Experimental Animal Center of Tsinghua University. They were placed in a quiet, temperature (23±3°C) and humidity (60±5%) controlled room with a 12∶12 hours light-dark cycle (light beginning at 8 a.m.). This study was conducted in accordance with the Guide for the Care and Use of Laboratory Animals of the China National Institutes of Health.

### Ischemia/reperfusion Injury Experimental Protocol

The acute myocardial I/R injury model was performed as previously described [25]. Male SD rats were anesthetized with pentobarbital sodium (30 mg/kg, i.p.). After a tracheotomy had been performed, rats’ lungs were ventilated mechanically with positive pressure ventilation using 30–40% air/oxygen mixture to maintain arterial blood gas pH within a physiological range by adjusting the respiratory rate and tidal volume throughout the experiment. Myocardial infarction (MI) was created by ligation of the left anterior descending (LAD)**.** The thorax was opened at the fourth or fifth left intercostal space. After left thoracotomy and pericardiotomy, MI was induced by LAD ligation 2–3 mm from the origin with a 6–0 silk suture. All animals (except for the rats in the sham groups) were subjected to 40 min of regional myocardial ischemia followed by 120 min of reperfusion. To confirm isoflurane-induced APC, a minimal alveolar concentration of isoflurane of 1.0 (2.1%) was started at the end of the stabilization period and administered for 30 min, followed by 30 min of washout before coronary occlusion.

Rats were randomly assigned to one of the following groups subjected to different protocols: Sham group, non-ischemic control group of sham-operated rats; non-ischemic control group of sham-operated rats with isoflurane; I/R group with isoflurane; I/R group without isoflurane (n = 5, respectively). To evaluate the role of ALDH2 in isoflurane-induced APC, the direct activator of ALDH2, Alda-44 (40 µM) [18], was given 5 min prior to ischemia in the groups without and with isoflurane (n = 8, respectively), and the ALDH2 inhibitor, cyanamide (5 mM) [20], was given without and with isoflurane (5 min prior to isoflurane) (n = 8, respectively). To verify that PKCε participates in the phosphorylation of ALDH2, the PKCε inhibitor, PKCε v1–2 (1 µM), was given 5 min prior to ischemia without and with isoflurane (n = 8, respectively, 5 min prior to isoflurane).

After taking blood samples, the heart was removed and perfused with Langendorff apparatus for 10 min to wash out the blood. The coronary artery was re-occluded and Evans Blue was infused into the aortic root to label the normally perfused zone with a deep blue colour. The heart was sectioned into transverse slices, which were incubated with 1% trimethyl tetrazolium chloride (TTC), and photographed by a digital camera. Since TTC stains viable tissue a deep red colour, non-stained tissue was presumed to be infarcted. Area at risk (negative for Evans Blue) and infarct area (negative for TTC) were quantified using Imageproplus software (Version 4. 1, Media Cybernetics, LP, USA) and infarct size was expressed as percentage of the area at risk (infarct area/AAR)×100 (%).

### Levels of Lactate Dehydrogenase and Creatine Kinase-MB in Plasma

Serum CK-MB analysis is a widely used biomarker to detect cardiac injury. Proportionally greater serum CK-MB, relative to the total CK activity can evaluate acute myocardial injury [8]. Before removing the heart, 5 ml blood samples were taken. Serum was separated by centrifugation at 5000 g for 5 min on a tabletop centrifuge; the supernatant was stored in liquid nitrogen. The samples were thawed for analysis. Lactate dehydrogenase (LDH) and creatine kinase-MB (CK-MB) were assayed using commercial kits (Roche, Germany) by an automatic analyzer 7600 (Hitachi, Japan).

### Western Blotting Analysis

Upon completion of the experimental period, the myocardium and cardiomyocytes were lysed in ice-cold radioimmunoprecipitation assay (RIPA) lysis buffer containing 1 mmol/L phenylmethylsulfonyl fluoride (PMSF), 1 µg/ml leupeptin, 1 µg/ml aprotinin and 1 µg/ml pepstatin at 4°C for 15 min. The homogenate was incubated and centrifuged. The supernatant was collected and the protein concentration was determined using the bicinchoninic acid (BCA) protein assay kit according to the manufacturer's protocol (Pierce). The detergent soluble supernatant was frozen with liquid N_2_, and stored at −70°C.

The supernatant was mixed with 5× loading buffer and heated for 5 min at 100°C. Soluble extracts (50 µg) were loaded in each lane and separated by SDS-polyacrylamide gel electrophoresis (PAGE). After electrophoresis, proteins were electrophoretically transferred to a polyvinylidene difluoride (PVDF) filter membrane (0.45 µm, Gehealthcare). The membrane was blocked in Tris-buffered saline Tween-20 (TBST) with 5% non-fat milk and incubated overnight with the corresponding primary antibodies at 4°C. The membrane was then incubated for 1 h with secondary antibody (horseradish peroxidase-conjugated antirabbit IgG) diluted with TBST (1∶2000). The signals of detected proteins were visualized by an enhanced chemiluminescence reaction (ECL) system (Millipore, Billerica, MA, USA). The staining was quantified by scanning the films and the band density was determined with Image-Pro software.

### Adenovirus Construction and Infection

Previous studies [18], [26] demonstrated that the constitutively active ALDH2 amino acid 487 must be Glu not Lys, and Thr185, Thr412 and Ser 279 must be constitutively phosphorylated. Accordingly, we obtained constitutively active mutant ALDH2 (CA-ALDH2) by nucleotide substitutions leading to the mutations Lys487Glu, Thr185Asp, Thr412Asp, and Ser279Asp introduced into the wild-type rat Aldh2 cDNA.

Short RNA hybrids (siRNAs) of 19 bp were formed by annealing two 21-mer oligoribonucleotides (Eurogentec, Belgium), each having two thymidines at their 3′ end. Rat-Aldh2 siRNA sequence was GCAACCAGATTCATTAATT [27]. The sense and antisense oligonucleotides were incubated together (1.5 nmol each) in 75 µL of 50 mM Tris (pH 7.5) and 100 mM NaCl for 2 min at 94°C, 5 min at 78°C and 5 min at 65°C. Finally, the annealed siRNAs were cooled to 20°C, aliquoted, and stored at −80°C. The cooling transitions was carried out at a rate of 2°C/min.

Viral vectors that expressed RFP, si-ALDH2 and RFP, the constitutively active mutant of ALDH2 (CA-ALDH2), and CA-ALDH2 and RFP were generated using the AdEasy system (Stratagene) [23]. Cardiomyocytes were prepared from ventricles and cultured in 60-mm dishes at a density of 1×10^5^ cells/cm^2^ in NCS-DMEM. After 24 h incubation at 37°C and 5% CO^2^, cell density reached approximately 70%. Cells were cultured overnight in 10% FBS-containing medium and infected with adenovirus for 6 h at a multiplicity of infection (MOI) of 20, then cultured in serum-free medium for an additional 24 h, before the addition of reagents.

### Cell Culture and Hypoxia/reoxygenation Treatment

Hearts were obtained from one-day old neonatal Sprague–Dawley rats, retaining the ventricles only, and kept in cold PBS without Ca^2+^ and Mg^2+^ on ice. The ventricles were rapidly minced and dissociated with 0.1% trypsin enzyme solution. The cells released after the first digestion were discarded, whereas the cells from subsequent digestions were added to NCS-DMEM (DMEM supplemented with 20% NCS, 100 U/ml penicillin, and 100 µg/ml streptomycin). After stepwise trypsin dissociation (10 min, 4–5 times), the mixture was centrifuged (1500 r/m, 5 min). The cells were resuspended in NCS-DMEM and first transferred to tissue culture dishes for 1 h in a 37°C incubator to plate out the fibroblasts [28]. The suspended cells were then replated at a density of 1×10^4^ cells/cm^−2^ and incubated under the same conditions as above. Bromodeoxyuridine (BrdU, 0.1 mM) was added to the medium for the first 2 days after plating to inhibit the growth of fibroblasts.

Simulated I/R was achieved by culturing the cells in 0.5% FBS DMEM in a hypoxia chamber, saturated with 5%CO_2_/95%N_2_ and supplemented with an anaerobic pouch (Mitsubishi Gas Chemical Company, Inc.) at 37°C for 24 h and following reoxygenation for 12 h using 0.5% FBS DMEM in the normal incubating condition [29]. Exposure to isoflurane was carried out by incubating the cells for 5 min in 0.5 mM isoflurane (approximately 1.0 minimum alveolar concentration) in 0.5% FBS DMEM. The isoflurane-containing medium was removed immediately before the onset of hypoxic conditions and the cells were washed with phosphate-buffered saline (PBS) [9]. Anesthetic concentrations were measured by gas chromatography (Gas chromatograph GC-8A; Shimadzu, Kyoto, Japan). Cells were grouped as follows: vector-infected with and without isoflurane, Adeasy-Si-ALDH2-treated with and without isoflurane; vector-infected with and without isoflurane, Adeasy-CA -ALDH2-treated with and without isoflurane.

### Apoptosis Assay

To determine cardiomyocyte apoptosis in a quantitative manner, the in situ detection of apoptotic cardiomyocytes was performed using terminal deoxyribonucleotide transferase-mediated dUTP nick end labeling (TUNEL) with an in situ cell death detection kit, Fluorescein (Roche, Germany) according to the manufacturer’s protocol for cultured cells. Cells (10^5^ cells/ml) from different treatment groups were cultured in a 6-well chamber slide and fixed in 4% paraformaldehyde followed by digestion with proteinase K (10 µg/ml) for 15 min at 37°C and permeabilization with 0.1% Triton X-100 for 5 min at 4°C. After washing twice with PBS, the cardiomyocytes were incubated with 50 µl TUNEL reaction mixture that contains TdT and fluorescein-dUTP for 1 h at 37°C. The percentage of TUNEL positive cells was determined by randomly chosen fields in each slide. In each group, at least 500 cells were counted. Sample evaluation was performed in a blinded manner, and samples from 3 independent experiments were scored per group.

### Measurement of Caspase 3 Activity

The Caspase 3 Colorimetric assay kit (MBL, MA, USA) was used to measure the activity of caspase 3 according to the manufacturer’s protocol. Cells were grown in a 6 well plate. After the appropriate treatment, cells were resuspended in lysis buffer and centrifuged. The supernatant was diluted with 50 ul cell lysis buffer for each assay. Then, the reaction buffer containing DTT and DEVD-pNA substrate were added to each assay and incubated at 37°C for 2 hours. After the correct incubation time, each sample was transferred to each well in a 96 well plate, and read at 405 nm using a microplate reader. Cell lysates were also analyzed by Western blotting with an antibody (Cell Signaling, Beverly, MA, USA) which allowed detection of inactive procaspase 3 and activated cleaved caspase 3.

### Statistical Analysis

Continuous values are expressed as mean ± standard error of the mean (SEM). Comparisons between multiple-group means were performed using one-way analysis of variance (one-way ANOVA) and comparisons between groups were performed using the least significant difference test (LSD-test). The number of animals/group and statistical significance for all data are listed in the figures and figure legends. P values <0.05 were considered to be statistically significant. All statistical analyses were performed using SPSS version 15.0.

## Results

### Isoflurane Preconditioning Attenuated the Release of LDH and CK-MB and Reduced Infarct Size in vivo I/R Injury

Regional myocardial ischemia for 40 min by LAD ligation followed by 120 min of reperfusion markedly increased the leakage of LDH (Figure 1A) and CK-MB (Figure 1B) compared to sham controls. Isoflurane-induced APC significantly reduced the I/R-induced increase in LDH and CK-MB release in rat heart.

**Figure 1:** The influence of anesthetic-induced preconditioning with 1.0 MAC of isoflurane on leakage of LDH and CK-MB, and infarct area in rat hearts. A, B. Serum LDH and CK-MB concentrations were analyzed. The increase in LDH and CK-MB concentrations was lower in rats pretreated with isoflurane than in I/R group. C. Isoflurane preconditioning significantly decreased infarct area compared with I/R group animals. Representative cross-sectional slices derived from a single heart with and without isoflurane. The infarct size normalized to the area at risk. Values are means ± S.E.M., n = 5 in each group. *P<0.05, **P<0.01 vs. sham group, and ^#^P<0.05 vs. the I/R control group.

As shown in Figure 1C, regional myocardial ischemia for 40 min by LAD ligation followed by 120 min of reperfusion significantly increased myocardial infarct size compared with sham groups. Isoflurane preconditioning substantially decreased I/R-induced myocardial infarct size.

### Phosphorylation of ALDH2 Participated in Cardioprotection Induced by Isoflurane Pretreatment

Representative gels for the different treatment groups are shown in Figure 2Aa. Figure 2Ab summarizes the quantitative data on the ratio of phosphoALDH2 to total ALDH2, and shows that pretreatment with isoflurane prior to ischemia increased the phosphorylation of ALDH2. The ALDH2 inhibitor, cyanamide, significantly inhibited isoflurane-induced activation of ALDH2. The direct activator of ALDH2, Alda-44, substantially increased the phosphorylation of ALDH2, but did not enhance the phosphorylation of ALDH2 by isoflurane.

**Figure 2:** Phosphorylation of ALDH2 associated with isoflurane-induced cardioprotection. A. Effects of isoflurane preconditioning with and without the ALDH2 inhibitor (cyanamide), and direct activator of ALDH2 (Alda-44) on phosphorylation of ALDH2. (a) Representative of western blot analysis of the phosphorylation of ALDH2 (phos-ALDH2 top lanes) and total ALDH2 (middle lanes). β-actin (lower lanes) was used to demonstrate equal protein loading. (b) Quantification of phos-ALDH2 to the total ALDH2 from 3 independent experiments. B, C. Serum LDH and CK-MB concentrations were analyzed. D. The effects of ALDH inhibitor (cyanamide), and direct activator of ALDH2 (Alda-44) on infarct area in rat hearts. (a) Representative cross-sectional slices derived from a single heart. (b) The infarct size normalized to the area at risk. Values are means ± S.E.M., n = 8 in each group.^ ##^P<0.01 vs. the saline control group and *P<0.05, **P<0.01 vs. the corresponding control.

Consistent with ALDH2 phosphorylation, we observed that isoflurane and Alda-44 markedly attenuated I/R-induced leakage of LDH and CK-MB in plasma, as well as myocardial infarct size. However, the isoflurane-induced decrease in LDH and CK-MB release, and reduction of infarct size was significantly blocked by the ALDH2 inhibitor cyanamide (Figure 2B–D). These findings suggest that isoflurane-mediated cardioprotection is mainly mediated by activation of ALDH2.

### Isoflurane Preconditioning Alleviated in vitro H/R Injury by Activation of ALDH2

To further confirm the critical role of ALDH2 in isoflurane-induced cardioprotection, we constructed an ALDH2 knockdown adenovirus and constitutively active ALDH2 mutant adenovirus. We used TUNEL, caspase 3 activity, and LDH release as quantitative assays to determine the functional significance of manipulating ALDH2 expression.

After 24 h of hypoxia followed by 12 h of reoxygenation we observed significant cardiomyocyte apoptosis demonstrated by increased DNA fragmentation using TUNEL staining, by laser scanning cytometry (LSC;) and caspase 3 activity in the vector control group. Pretreatment with isoflurane significantly inhibited the H/R-induced increase in TUNEL positive staining, caspase 3 activity and leakage of LDH (Figure 3B–E). However, when ALDH2 was downregulated (Figure 3A) in cardiomyocytes by Ad-Si-ALDH2, increased TUNEL positive staining level (Figure 3B), more intense cleaved caspase-3 staining (Figure 3C), caspase 3 activity (Figure 3D) and LDH release (Figure 3E) were observed, which supports the hypothesis that phosphorylation of ALDH2 might play a critical role in isoflurane-induced cardioprotection. Immunoblotting analysis showed a substantial increase in ALDH2 level in Ad-CA-ALDH2-RFP-infected cells compared to Ad-RFP (Figure 4A). Constitutively active ALDH2 significantly inhibited the H/R-induced increase in TUNEL positive staining, caspase 3 activity and leakage of LDH (Figure 4 B–E), which were not further increased by isoflurane treatment.

**Figure 3:** ALDH2 knockdown blocks isoflurane-induced protection against hypoxia/reoxygenation. A. Schematic representation of adenoviruses encoding RFP (Ad-RFP) and ALDH2shRNA (Ad-Si-ALDH2-RFP, left panel); right panel, immunoblotting analysis of ALDH2 protein level. β-actin was used as a control. B. ALDH2 down-regulation inhibited attenuation of TUNEL positive staining level by isoflurane. (a) Apoptotic cells were examined using TUNEL assay for DNA fragmentation. Cardiomyoctes were photographed by fluorescence microscopy after 24 hours of hypoxia followed by 12 hours of reoxygenation. TUNEL-positive nuclei are shown in green and transfection efficiency of adenoviruses in red. (b) Quantitative analysis (percentage of apoptotic cells versus total) is shown in histogram. C. Representative Western blots of cleaved caspase-3 and full length caspase-3 (FL caspase-3) in (a), and 3 independent experiments were quantitated in (b). β-actin was used as a loading control. D. Cell lysates under each condition were quantitatively assayed for caspase-3 activity. E. LDH concentrations in cell culture media were analyzed. Values are means ± S.E.M., n = 5 in each group. *P<0.05, **P<0.01 vs. Control group, and ^#^P<0.05, vs. the corresponding Ad-RFP group.

**Figure 4:** ALDH2 activation induced protection against hypoxia/reoxygenation. A. Schematic representation of adenoviruses encoding RFP (Ad-RFP) and CA-ALDH2 (Ad-CA-ALDH2-RFP, left panel); right panel, immunoblotting analysis of ALDH2 protein level. β-actin was used as a control. B. Expression of constitutively active mutant of ALDH2 attenuated TUNEL positive staining level, which was not reinforced by isoflurane. (a) Apoptotic cells were examined using TUNEL assay for DNA fragmentation. Cardiomyoctes were photographed by fluorescence microscopy after 24 hours of hypoxia followed by 12 hours of reoxygenation. TUNEL-positive nuclei are shown in green and transfection efficiency of adenoviruses in red. (b) Quantitative analysis (percentage of apoptotic cells versus total) is shown in histogram. C. Representative Western blots of cleaved caspase-3 and FL caspase-3 in (a), and 3 independent experiments are quantitated in (b). β-actin was used as a loading control. D. Cell lysates under each condition were quantitatively assayed for caspase-3 activity. E. LDH concentrations in cell culture media were analyzed. Values are means ± S.E.M., n = 5 in each group. *P<0.05, **P<0.01 vs. Control group, and ^#^P<0.05 vs. the corresponding Ad-RFP group.

### PKCε is Involved in Isoflurane-induced Phosphorylation of ALDH2 and Cardioprotection

PKCε translocation to mitochondria and then phosphorylation of ALDH2 is required to protect the heart from I/R injury. Here we demonstrate that pretreatment with isoflurane resulted in elevated mitochondrial levels of PKCε accompanied by phosphorylation of ALDH2. Isoflurane-induced phosphorylation of ALDH2 was inhibited by the PKCε inhibitor, PKCε V1–2. Because mitochondrial translocation of PKCε occurs rapidly, with a corresponding decline in cytosolic PKCε levels, and because the total cellular PKCε levels do not change (Figure 5A), our data suggest that isoflurane enables dynamic mitochondrial translocation of PKCε in response to I/R. Consistent with PKCε translocation to mitochondria, PKCε V1–2 had a detrimental effect on isoflurane-induced attenuation of LDH and CK-MB leakage (Figure 5B, 5C), and the decrease in myocardial infarct size (Figure 5D).

**Figure 5:** PKCε translocation is involved in isoflurane preconditioning. A PKCε translocation was associated with isoflurane-induced phosphorylation of ALDH2. (a) Representative of western blot analysis of phos-ALDH2, total ALDH2, β-actin, mitochondria PKCε (mito-PKCε) and total PKCε (from top lanes to bottom lanes). β-actin was used to demonstrate equal protein loading. (b) Quantification of the phos-ALDH2, normalized to the total ALDH2, and PKCε translocation to the mitochondria from 3 different experiments. B, C. Isoflurane-induced inhibition of LDH and CK-MB release by I/R was restored by PKCε v1–2. Serum LDH and CK-MB concentrations were analyzed. D. PKCε v1–2 inhibits the decrease in heart infarct size caused by isoflurane following I/R. Representative cross-sectional slices derived from a single heart. The infarct size normalized to the area at risk. Values are means ± S.E.M., n = 8 in each group. *P<0.05, **P<0.01 vs. the saline control group and ^#^P<0.05, ^##^P<0.01 with PKCε v1–2 vs. the corresponding group without PKCε v1–2.

## Discussion

In the present study, we observed that (1) isoflurane pretreatment reduced I/R injury in vivo and stimulated H/R insult in vitro associated with phosphorylation of ALDH2; (2) isoflurane-induced phosphorylation of ALDH2 and cardioprotection was mediated by PKCε translocation from the cytosol to mitochondria. Thus, phosphorylation of ALDH2 is critical for the cardioprotective effects of isoflurane preconditioning.

Volatile anesthetics have a long history in the clinical management of anesthesia. Consistent with our results, numerous studies have shown that volatile anesthetics can protect the myocardium when applied before a harmful ischemic event and at the beginning of reperfusion, and that the characteristics of this protection are similar to those observed during classic IPC. Studies have attempted to characterize the mechanisms involved. Cardioprotective mechanisms produced by APC were shown to involve activation of phosphoinositide 3-kinase [25], extracellular regulated kinases 1 and 2 (ERK1/2) [30], the 70-kDa ribosomal protein S6 kinase, endothelial ROS (eNOS) [31], mitochondrial K_ATP_ channels [3], [14], [15] and inhibition of glycogen synthase kinase 3-β [32], but the precise mechanism responsible for APC remains undefined. However, it is unlikely that stimulation of pro-survival signaling pathways occurs rapidly enough to prevent damage resulting from the initial injury during reperfusion. Recently, attention has focused on mitochondria as a target of cardioprotection by volatile anesthetics [11], [33], [34].

Mitochondria are essential for cell survival and play important roles in the complex signaling pathways leading to cardioprotection by volatile anesthetics, and in the production of adenosine triphosphate and the regulation of cell death [35]. The mechanisms by which isoflurane ultimately limits infarct size are not known. Apoptosis and inflammation have been implicated in cardiac I/R injury [36]–[39]. In agreement with our results, isoflurane-treated mice subjected to ischemia and 2 weeks of reperfusion showed reduced expression of proapoptotic genes, significantly decreased expression of cleaved caspase-3, and TUNEL staining [5].

ALDH2 is best known for its role in metabolizing the ethanol intermediate, acetaldehyde. These highly toxic, reactive aldehydes can create aldehydic adducts with proteins, causing protein dysfunction and tissue injury, and have been linked to various diseases, such as cancer and MI, in humans [40]. It has been reported that overexpression of the ALDH2 transgene may alleviate I/R injury, post-I/R and ischemic ventricular dysfunction [21], [41]. Consistent with this, I/R injury may be exacerbated by ALDH2 knockout [23], [41]. These data support our results that ALDH2 plays an essential role in isoflurane-induced cardioprotection against I/R injury. It was shown that overexpression of ALDH2 significantly attenuated acetaldehyde and ethanol-induced oxidative stress (ROS generation), activation of stress signal molecules and apoptosis in fetal human cardiac myocytes [21]. Here, we showed that isoflurane preconditioning increased the phosphorylation of ALDH2. These data also support our notion that isoflurane pretreatment attenuated I/R-induced apoptosis which is associated with phosphorylation and activation of ALDH2.

We observed that isoflurane pretreatment led to PKCε translocation to mitochondria. Although phosphorylation and translocation of PKC are thought to be pivotal steps in cardioprotection by IPC, and PKCε seems to play a critical role in the signaling cascade underlying preconditioning [11], [16], there are few data suggesting the involvement of PKC in APC [11], [42]. It has been shown that phosphorylation and translocation of PKCε depends on the concentration of the volatile anesthetic and that alternative pathways may exist at higher concentrations [30]. Recent studies reported that PKCε targeted the inner mitochondrial membrane and phosphorylated a number of intra-mitochondrial proteins [18], [43], [44]. Mitochondrial ALDH2 has been identified as a PKCε substrate, whose activity correlates with cardioprotection against I/R [18], [20]. Our results showed that isoflurane-induced ALDH2 activation was accompanied by translocation of PKCε from the cytosolic to the mitochondria fraction, which was inhibited by the PKCε inhibitor. It was shown that ERK1/2 blockade abolished PKCε activation, suggesting ERK pathway was involved in activation of PKCε, during desflurane-induced preconditioning [30]. Opening of mitochondrial adenosine triphosphate-sensitive potassium channels and generation of reactive oxygen species were upstream events of PKCε activation in isoflurane-induced preconditioning [45]. Activation of ALDH2 can attenuate ROS production [21], indicating that ALDH2 might be a critical mediator of isoflurane-induced protection. Further research needs to be carried out to identify the ALDH2 mechanism in mitochondria.

Although polymorphism in ALDH2 gene is an independent risk factor for myocardial infarction [46], [47], a recent study showed that inhibited ALDH2 activity during cardiac surgery got less I/R injury and better cardiac function [48]. The contradicted clinical results might need larger sample and stronger evidence to testify. However, from point of view of clinical application of APC in the future, in patients with lower Aldh2 activity who experience an ischemic event, the use of isoflurane may need to be reconsidered.

In summary, our results demonstrate that isoflurane preconditioning increased the phosphorylation of mitochondrial ALDH2 which was mediated by mitochondrial PKCε and is required for cardiac protection against I/R (Figure 6). This work suggests a possible mechanism by which isoflurane can access cytoprotective substrates located within the mitochondria to confer cardioprotection [49]. Our data provide an insight into the mitochondrial-dependent basis of isoflurane-induced, and PKCε and ALDH2-mediated protection against cardiac ischemia, in vivo and in vitro [19]. The current study extends our understanding of APC cardiac protection, which is relevant for extrapolation to the clinic.

**Figure 6:** Hypothetical scheme demonstrate that the phosphorylation of ALDH2 through mitochondrial translocation of PKCε plays an important role in the cardioprotection of isoflurane preconditioning in myocardium I/R injury. Ischemic preconditioning/postconditioning and pharmacological agents result in the activation of the RISK pathway, which lead to the phosphorylation and mitochondrial translocation of PKCε.
